The article "Epidemiological Pattern of Newly Diagnosed Children with Type 1 Diabetes Mellitus, Taif, Saudi Arabia" was retracted in 2016. Reasons: plagiarized text; content taken from a thesis; overlap with other authors' work; concerns about the citations.

# Epidemiological Pattern of Newly Diagnosed Children with Type 1 Diabetes Mellitus, Taif, Saudi Arabia

**DOI:** 10.1155/2013/421569

**Published:** 2013-10-09

**Authors:** Naglaa Mohamed Kamal Alanani, Adnan Amin Alsulaimani

**Affiliations:** ^1^Pediatric Department, Faculty of Medicine, Cairo University, Cairo, Egypt; ^2^Pediatric Department, Faculty of Medicine, Taif University, Saudi Arabia

## Abstract

*Introduction and Aim.* Type-1-diabetes mellitus (T1DM) is the most commonly diagnosed type of DM in children and adolescents. We aim to identify the epidemiological profile, risk factors, clinical features, and factors related to delayed diagnosis or mismanagement in children with newly diagnosed T1DM in Taif, Saudi Arabia. *Patients and Methods.* Ninety-nine newly diagnosed patients were included in the study along with 110 healthy controls. Patients were classified into 3 groups (I: >2 years, II: 2–>6 years, and III: 6–12 years). Both patients and controls were tested for C-peptide, TSH, and autoantibodies associated with DM and those attacking the thyroid gland. *Results*. Diabetic ketoacidosis was present in 79.8%. Delayed and missed diagnoses were recorded in 45.5%, with significant correlation to age and district of origin. Severity at presentation showed significant correlation with age and cow's milk feeding. Group I, those with misdiagnosis or positive DM related autoantibodies, had more severe presentations. The correlation of C-peptide and TSH levels in patients and controls was significant for C-peptide and nonsignificant for TSH. *Conclusion. *Misdiagnosis and mismanagement are common and account for more severe presentation, especially in young children >2 years. Early introduction of cow's milk appears to be a risk factor for the development of T1DM.

## 1. Introduction

Type 1 diabetes mellitus (T1DM) is the most commonly diagnosed type of DM in children and adolescents. It presents usually with symptomatic hyperglycemia and imparts the immediate need for exogenous insulin replacement [1].

The presentation of T1DM is either as classic new onset DM (most common), silent DM, or diabetic ketoacidosis (DKA) which constitutes 20%–40% of cases [2].

The classic new onset T1DM patients present with polyuria, polydipsia, polyphagia, weight loss, and lethargy, while those with silent T1DM are typically diagnosed by families or physicians with high index of suspicion. Children who present with DKA also present with dehydration, vomiting, altered mental status, and rapid deep respiration (Kussmaul's breathing) [3]. 

Because DKA is a potentially preventable acute complication of DM and a predominant cause of mortality in children with diabetes, early recognition and prompt treatment should substantially reduce mortality in children with T1DM [4].

The article "Epidemiological Pattern of Newly Diagnosed Children with Type 1 Diabetes Mellitus, Taif, Saudi Arabia" was retracted in 2016. Reasons: plagiarized text; content taken from a thesis; overlap with other authors' work; concerns about the citations.

Increased public awareness of early symptoms of diabetes is needed to reduce the incidence and severity of DKA. In addition, greater medical alertness to the possibility of T1DM in a young child should be stressed [5].

The aim of the present study is to identify the main epidemiological patterns, clinical features, and risk factors for newly diagnosed children with T1DM in Taif district, Saudi Arabia. We aimed also at identification of the risk factors related to delayed diagnosis or mismanagement of newly diagnosed patients.

## 2. Patients and Methods

### 2.1. Patients

We carried a prospective study during the period from March 2011 to March 2013 on ninety-nine Saudi children with newly diagnosed T1DM aged from birth to twelve years old from those attending the Pediatric Endocrinology outpatient clinics, the Pediatric Emergency units and the Pediatric inpatients wards, Taif region Hospitals, Saudi Arabia. One hundred and ten healthy children of matched age and sex from those attending the Well Child clinics served as controls.

Written informed consents were obtained from all patients' and controls' parents for contribution into the current study. The study was approved by the research and ethical committees of the contributing hospitals.

### 2.2. Methods

Patients were classified according to age into 3 groups ((I): <2 years, (II): 2–<6 years, and (III): 6–12 years). All patients were subjected to the following.

- *Full history taking:* age, district of origin, mode of presentation, clinical symptoms preceding diagnosis, duration before diagnosis, delayed or misdiagnosis, associated endocrinopathies or autoimmune diseases at onset, nutritional history at infancy (breastfeeding, cow's milk feeding whether formulas, yogurt, or other milk derivatives), family history including consanguinity, and positive family history of diabetes, other endocrinopathies or autoimmune diseases.
- *Thorough clinical examination: *anthropometric measurements obtained following the recommendations of the international biological program [6] and plotted on the Saudi children growth charts [7], thorough general and body systems examination [8].
- *Classification:* DKA categorization was carried according to the American Diabetes Association into three stages of severity [9].
  - Mild: blood pH mildly decreased to between 7.25 and 7.30 (normal 7.35–7.45); serum bicarbonate decreased to 15–18 mmol/L (normal above 20); the patient is alert.
  - Moderate: pH 7.00–7.25, bicarbonate 10–15, mild drowsiness may be present.
  - Severe: pH below 7.00, bicarbonate below 10, stupor or coma may occur.
- *Laboratory investigations*: all patients were tested at initial presentation for blood glucose, urine acetone, blood gases, serum electrolytes, kidney functions, thyroid stimulating hormone (TSH), autoantibodies associated with DM (insulin autoantibodies (IAA) and glutamic acid decarboxylase antibodies (GADA), islet cells antibodies (ICA)), and autoantibodies to the thyroid gland. After stabilization and an overnight fasting (>6–8 hours), patients were tested for fasting blood sugar and fasting C-peptide.

The article "Epidemiological Pattern of Newly Diagnosed Children with Type 1 Diabetes Mellitus, Taif, Saudi Arabia" was retracted in 2016. Reasons: plagiarized text; content taken from a thesis; overlap with other authors' work; concerns about the citations.

All controls were tested for fasting blood sugar, fasting C-peptide, TSH, and autoantibodies associated with DM and those against thyroid gland.

## 3. Statistical Methods

- Data management and analysis were performed using Statistical Analysis Systems, SAS versus 8.02.
- Numerical data were summarized using means and standard deviations or medians and ranges. Categorical data were summarized as percentages. Differences between two groups with respect to numeric variables were tested using the Student's *t*-test or Mann-Whitney, for small sample size. A one-way analysis of variance for small sample size, Kruskall-Wallis test, was performed to test differences between more than two groups. Chi-square test was used to compare groups with respect to categorical data or Fisher's exact test, for small sample size [10].
- All *P* values are two sided. *P* values < 0.05 were considered significant.

## 4. Results

Ninety-nine children, 52 males (52.5%) and 47 females (47.5%), with newly diagnosed T1DM were included in the current study. The mean age at diagnosis was 6.8 years ±4.6 (range 0.39–12 years) in males and 6.6 ± 4.2 years (range 0.19–12 years) in females. Patients were classified according to age into 3 groups ((I): <2 years, (II): 2–<6 years, and (III): 6–12 years). The demographic data of the studied population are shown in Table 1. 

Sixty percent of patients were coming from rural areas and 40% from urban areas. They were distributed more or less similarly among the three age groups with *P* > 0.05 (Table 1). 

The main symptoms preceding the diagnosis are illustrated in Figure 1 where polyuria, polydipsia, and weight loss (the classic triad of DM) had the highest percentage followed by nocturia and nocturnal enuresis then abdominal pain follows.

Disturbed conscious level was present in an appreciable percentage (46.5%) being more frequent in those <2 yrs (60.9%) compared to 40.9% and 42.6% in group II and III, respectively.

The distribution and correlation of the main symptoms experienced by the patients prior to diagnosis with the studied age groups are shown in Table 2 where polyphagia was found to be more frequent than decreased appetite and refusal of feeding (Figure 1), with no age differences.

The article "Epidemiological Pattern of Newly Diagnosed Children with Type 1 Diabetes Mellitus, Taif, Saudi Arabia" was retracted in 2016. Reasons: plagiarized text; content taken from a thesis; overlap with other authors' work; concerns about the citations.

Abdominal pain was found more frequent as the age gets older. Around 14.3% of those below 2 years had colics and refusal of feeding, while 40.9% and 74% of both groups II and III, respectively, had abdominal pain with a statistically significant higher frequency in the 6–12 years age group (*P* < 0.001). Nocturia and nocturnal enuresis were found to be more frequent in group III with *P* < 0.001.

Most patients presented with moderate to severe DKA (51.5%), followed by mild DKA in 28.3%. Only 20.2% presented with hyperglycemia without ketoacidosis. The correlation between the mode of presentation and age is shown in Table 1, where those <2 years presented more severe.

The majority of the cases with abdominal pain (84.6%) presented with DKA at diagnosis, being moderate to severe in 2/3. All cases complaining of vomiting at diagnosis were in DKA, again being moderate to severe in 2/3. The triad of abdominal pain, vomiting, and dehydration were evident in all cases presenting with moderate to severe DKA (Table 3).

The duration of symptoms before diagnosis varied greatly in such way that the standard deviation was found to be greater than the mean itself, accordingly we preferred the median which was found to be 14 days (range 1 to 180 days), as shown in Table 1.

There was a significant correlation between the duration of symptoms and the districts of origin with higher duration of symptoms among those coming from rural areas, *P*  value = 0.028 (Figure 2).

Twelve patients had prolonged duration of symptoms before diagnosis. Eight patients had 60 days duration; 5 of them presented to us with moderate to severe DKA, and the other 3 presented with mild DKA. Two patients (4 months and 1.6 years) presented after 90 days duration of symptoms with hyperglycemia and mild DKA, respectively. They were misdiagnosed as gastroenteritis (GE) and weaning problems, respectively.

One child, 11 years, had 140 days duration of symptoms. He presented with moderate to severe DKA and was misdiagnosed as GE.

The child with the longest duration of symptoms, 180 days, presented with hyperglycemia only and had delayed diagnosis due to atypical symptoms (headache, nausea, and abdominal pain).

The severity of presentation at the time of diagnosis among the different age groups is presented in Table 1, which shows that 20 children (20.2%) presented with hyperglycemia without ketosis, 28 (28.3%) with mild DKA, and 51 (51.5%) with moderate to severe DKA. Group I and III presented more severe with moderate to severe DKA (*P* < 0.05) (Table 1). 

High percentage of the studied population (45.5%) were misdiagnosed at their initial presentation. They were misdiagnosed either as upper (25%) or lower (37.5%) respiratory tract infection, or gastroenteritis (37.5%). Misdiagnosis was found to be statistically higher in group I as compared to the other 2 groups (69.6% versus 36.4 and 38.9%, *P* < 0.05) (Table 1) with a higher percentage of misdiagnosis among those living in rural areas (Figure 3).

The article "Epidemiological Pattern of Newly Diagnosed Children with Type 1 Diabetes Mellitus, Taif, Saudi Arabia" was retracted in 2016. Reasons: plagiarized text; content taken from a thesis; overlap with other authors' work; concerns about the citations.

Regarding family history (FH) of DM, it was found that positive FH of type-2-DM (T2DM) only was more common in the three age groups as compared to FH of T1DM only or to both T1DM and T2DM (Table 1).

Analysis of the type of feeding in the studied population revealed that only 19 patients were absolutely breastfed while 80 patients were cow's milk fed (Table 4).

The median duration of breastfeeding in the study population was 1.5 years, range from zero (no breastfeeding) to 2 years. The duration of breastfeeding in the absolutely breastfed group was 0.68–2 years. Among them, 17 (89.5%) had positive FH of diabetes; 9 with T2DM; and 8 with both T1DM and T2DM but among them only 4 had the positive FH of DM in a first degree relative.

Early introduction of cow's milk was classified according to the time of introduction into 3 subclasses: <3 months (28, 28.3%), 3–6 months (24, 24.2%), and >6 months (28, 28.3%).

The relation between type of feeding and the age at presentation is illustrated in Figure 4 where the mean age of breastfed group was 6.8 years (range 0.1–12 yrs). The mean age for the 3 subgroups of cow's milk feeding (<3 months, 3–6 months, and >6 months) was 5.7 yrs (range 0.3–12 yrs), 6.5 yrs (range 0.9–12 yrs), and 7.6 yrs (range 0.6–12 yrs), respectively. Those who were cow's milk fed presented at earlier age, *P* value < 0.05.

Implications of different factors on the severity of diabetes presentation are studied in Figures 3 and 4. Figure 3, highlights that small children (<2 years), those with misdiagnosis, or positive antibodies to insulin and islet cells had more severe presentations as most of them presented with moderate to severe DKA. These antibodies were detected with statistically higher percentage in patients with moderate to severe DKA as compared to other groups, (*P* < 0.001). Table 4 showed that 80.8% of patients were cow's milk fed which could raise the issue of early cow's milk feeding as a risk factor for T1DM. It also showed a significant correlation between early introduction of cow's milk and the severity of presentation.

 Regarding family history, it was statistically insignificant in the three groups (Table 4), yet children having positive FH for DM had lower frequency of misdiagnosis as compared to those with negative FH. Twenty-four patients had FH of autoimmune disease, goiter in 20 and collagen vascular disease in 4.

The article "Epidemiological Pattern of Newly Diagnosed Children with Type 1 Diabetes Mellitus, Taif, Saudi Arabia" was retracted in 2016. Reasons: plagiarized text; content taken from a thesis; overlap with other authors' work; concerns about the citations.

Table 5 displays the correlation of C-peptide and TSH levels in patients and controls which was significant for C-peptide and nonsignificant for TSH. However, there was statistical variation in TSH levels and thyroid antibodies in the 3 studied patients groups with tendency to be higher in group III (Table 1).

Regarding consanguinity, all patients had positive consanguinity that is why the role of consanguinity cannot be judged.

## 5. Discussion 

The current study included 99 children with newly diagnosed diabetes who were classified according to age into 3 age groups ((I): <2 years, (II): 2–<6 years and (III): 6–12 years) with higher incidence of disease in the older age group which is in accordance with several authors [11–14] while the younger age groups showed a rising incidence (45.5% in <6 years) which was in agreement with Harjutsalo et al. [15] and Patterson et al., [16], who expected in their studies doubling of the incidence of T1DM over the next 10 years. The EURODIAB reported a very wide range of incidence rates within Europe with the greatest increase in incidence rate among the young age groups [16].

In the present study, 60% of patients came from rural areas and 40% from urban areas with a ratio of 1.4 : 1. In agreement with other studies [17], the classic triad of DM were the most common symptoms preceding diagnosis in all age groups indicating that simple increased awareness of the necessity to consider diabetes in presence of this triad should improve recognition of diabetes with no delay in all age groups even infants.

Abdominal pain was more frequent as the age gets older specially the 6–12 years age group when the child can more reliably relay his symptoms. Increasing the awareness of the public and health care professionals about these symptoms as possible features of diabetes and the necessity of routine urine or blood glucose analysis when these symptoms are encountered can decrease the frequency and severity of DKA. Same applies to nocturia and nocturnal enuresis, which are considered reliable symptoms in those above 2 years. Roche et al. (2005) agreed with us in that respect [18].

Disturbed conscious level was present in an appreciable percentage signifying more severe presentation at time of diagnosis. It was more frequent in those below 2 yrs which relates to the delay in diagnosis and the severity of diabetes in this young age group.

Infants below 2 years of age showed the highest frequency of moderate to severe DKA (73.9%). This finding is in agreement with several studies [5, 19–23]. Neu et al. [19] and Szypowska and Skórka [23] suggested that children under 2 yrs of age remain the most prone to DKA due to delay in diagnosis as well as more aggressive *β*-cell destruction which is in agreement with the current study as seen from the highest incidence of misdiagnosis (Figure 2).

The article "Epidemiological Pattern of Newly Diagnosed Children with Type 1 Diabetes Mellitus, Taif, Saudi Arabia" was retracted in 2016. Reasons: plagiarized text; content taken from a thesis; overlap with other authors' work; concerns about the citations.

The median duration of symptoms before diagnosis was 14 days (range 1–180 days) which was significantly higher in rural compared to urban areas; Du Prel et al. [24] suggested that the risk for T1DM is higher in children living in socially deprived and less densely populated areas. In addition, our study attributed the significantly increased severity of symptoms at presentation also to misdiagnosis (Figure 2). Misdiagnosis was found in 45.5% of the included patients, with around 25% being misdiagnosed as upper respiratory tract infections, 37.5% as lower respiratory tract infections, and 37.5% as gastroenteritis. Misdiagnosis was found to be the cause of long duration and severe presentations with moderate to severe DKA. In Saudi Arabia, Rotavirus is considered the most common cause of childhood gastroenteritis [25, 26]; on the other hand, Honeyman et al. 2000 [27] reported that serologically defined Rotavirus infection is significantly associated with an increase in ICA levels, then with IAA and GADA. This could explain the high levels of these autoantibodies in the present study especially in cases with moderate to severe DKA.

A consensus statement from American Diabetes Association precisely points out delayed diagnosis as one of the main causes of DKA development in many children with newly diagnosed T1DM [28].

Regarding severity at presentation, it ranged from hyperglycemia to severe DKA. The frequencies of the different grades of severity were comparable between urban and rural areas. No significant difference was found in the duration of symptoms neither in relation to age nor to the degree of severity at presentation. This was similar to Olak-Białoń et al. [29], who found no correlation between duration of symptoms and both the severity of DKA and age of children.

In the present study, positive family history of T2DM was more frequent than type 1 or both, in the 3 age groups, which was in agreement with Barone et al. [30]. Unfortunately, the presence of positive FH did not improve recognition of diagnosis and did not decrease duration of symptoms nor severity at presentation in our cohort which was in contrary to Blanc et al. [31] who found significantly less frequency of DKA in children with positive FH of T1DM. This might point to the low awareness and sometimes to denial and high resistance of the families with a positive FH of DM to admit the fact that other family members are prone to the development of DM. This issue is a real actual obstacle which we faced in many patients which was very evident up to the stage that some parents of children who presented with DKA even the severe grade were highly reluctant to admit that their children had T1DM and a false fixed believe that this might be a transient event which will resolve. Another great obstacle which might be very unique is the great believe of parents in traditional herbal medicines and their false thinking that this type of medicine can treat their children without the use of insulin. All these issues highlight the great need to emphasize and stress on health education and awareness about DM especially for members of families with positive FH. A multidisciplinary approach with involvement of physicians, dietitians, nutritionists, health educators, diabetic educators, social workers, and psychiatrists is highly recommended.

The article "Epidemiological Pattern of Newly Diagnosed Children with Type 1 Diabetes Mellitus, Taif, Saudi Arabia" was retracted in 2016. Reasons: plagiarized text; content taken from a thesis; overlap with other authors' work; concerns about the citations.

An interesting finding in the current study which reflects the lack of awareness about healthy life style behaviors is the very low percentage of exclusively breastfed infants (19.2%) compared to 80.8% with cow's milk feeding which was introduced as early as <3 months age. Correlation of type of feeding with age at presentation revealed an earlier median age of around 4 years in children with early cow's milk introduction (<3 months) compared to an older median age of 7 years and 8 years in exclusively breastfed and late cow's milk introduction (>6 months), respectively. These findings may support the suggestions for the protective role of breastfeeding on one hand and the early cow's milk introduction as a risk factor for development of T1DM on the other hand. A review paper “Milk and Diabetes” [32] listed several studies which suggest that cow's milk products are associated with the onset of T1DM, and several other studies which show no correlation. The literature is still equivocal about the relationship of cow's milk products and the risk of type 1 diabetes, particularly the relationship between the time of their introduction to an infant and the onset of diabetes. Another review article [33] discussed this unsettled issue with several studies relating the age of introduction of dairy products to the risk of T1DM in particular when formula is introduced before 4 months of age, while other studies were not supporting this association. The same article added more evidence that cow's milk proteins trigger T1DM where antibodies to bovine beta-lactoglobulin were detected in the serum of children with diabetes while individuals without diabetes did not have this antibody [33]. According to a recent review article, most studies suggest that the early introduction of complex foreign proteins may be a risk factor for beta-cell autoimmunity, and a pilot intervention trial has implied that weaning to a highly hydrolyzed formula may decrease the risk of beta-cell autoimmunity [34]. Achenbach et al. 2005 [35] reported that children who develop autoantibodies within the first 2 years of life are those who most often develop multiple islet autoantibodies and progress to T1DM in childhood. This was very similar to the current study which revealed that most of cases below 2 years developed ICA, IAA, and GADA. Achenbach added that children who develop autoantibodies above 2 years have a slower progression to multiple antibodies and T1DM [35]. Kordonouri et al., 2002 [36], agreed with us in reporting significant prevalence of thyroid antibody titers with older age (Table 1). They added that TSH levels were higher in patients with thyroid autoimmunity [36]. Accordingly, the American Diabetes Association [37] and several authors [38, 39] recommended annual screening for thyroid disease in all T1DM subjects with TSH measurement; this procedure is considered the most sensitive way to identify patients with thyroid dysfunction, as autoantibodies may persist for many years without thyroid dysfunction.

The article "Epidemiological Pattern of Newly Diagnosed Children with Type 1 Diabetes Mellitus, Taif, Saudi Arabia" was retracted in 2016. Reasons: plagiarized text; content taken from a thesis; overlap with other authors' work; concerns about the citations.

Fasting C-peptide was done in all patients after stabilization at their initial presentation which ranged from 0.25 to 3.8 ng/mL (mean 1.07 and median 0.87 ng/mL) that was in agreement with Levitt Katz et al. [40] who reported fasting C-peptide levels 0.38 ± 0.37 ng/mL with 83% sensitivity in distinguishing T1DM from T2DM.

## 6. Conclusions

1. The classic triad (polyuria, polydipsia, and weight loss) is the commonest presenting symptom of diabetes in children. Misdiagnosis and mismanagement are common and account for more severe presentation among newly diagnosed children with diabetes, with those below 2 years of age being the most vulnerable group to such problem.
2. Early introduction of cow's milk feeding appears to be a risk factor for the development of T1DM but more studies with larger population are warranted to validate these results.
3. Increasing the awareness of the public especially in rural areas about the following:
  - the great benefit of absolute breastfeeding in the 1st 6 months of their babies' life;
  - the possibility of occurrence of DM in young children especially those with positive FH of DM and the better outcome when diagnosed early.
4. A multidisciplinary approach with involvement of physicians, dietitians, nutritionists, health educators, diabetic educators, social workers, and psychiatrists is highly recommended.

## Figures and Tables

**Figure 1:** Common symptoms preceding presentation and common signs at presentation in the studied group.

The article "Epidemiological Pattern of Newly Diagnosed Children with Type 1 Diabetes Mellitus, Taif, Saudi Arabia" was retracted in 2016. Reasons: plagiarized text; content taken from a thesis; overlap with other authors' work; concerns about the citations.

**Figure 2:** Duration of symptoms in relation to district in the studied group.

**Figure 3:** Risk stratification of severity of presentation of type I diabetes mellitus in the studied patients. Note that analysis of the severity of presentation in relation to the district of origin and age groups was statistically nonsignificant for those from urban areas (*χ*2 = 1.25, *P* > 0.05), but highly significant statistically for those from rural areas (*χ*2 = 16.4 and *P* = 0.0025), indicating that children living in rural areas had more severe presentation (moderate to severe DKA).

**Figure 4:** Relation between type of feeding and age at presentation in the studied patients.

**Table 1:** Demographic data of the studied patients.

Point of comparison	<2 years		2–<6 years		6–12 years		Total		*P* value
	No.	%	No.	%	No.	%	No.	%	
Number	23	23.2	22	22.2	54	54.4	99	100	—
District									
Urban	10	43.5	7	31.8	23	42.6	40	40	*P* > 0.05
Rural	13	56.5	15	68.2	31	57.4	59	60	
Symptoms duration									
(*X* ± SD)	21 ± 17.6		22 ± 22.5		27 ± 33.6				*P* > 0.05
Median	10		16		14			
Severity of presentation									
Hyperglycemia without DKA	4	17.4	5	22.7	11	20.4	20	20.2	*P* = 0.04
Mild DKA	2	8.7	10	45.5	16	29.6	28	28.3	
Moderate to severe DKA	17	73.9	7	31.8	27	50	51	51.5	
Misdiagnosis	16	69.6	8	36.4	21	38.9	45	45.5	*P* < 0.05
FH									
T1DM	1	4.7	0	0	2	3.7	3	3	*P* > 0.05
T2DM	15	71.5	13	59.1	29	53.7	57	57.6	*P* < 0.05
T1DM and T2DM	3	14.2	5	22.7	10	18.5	18	18.2	*P* > 0.05
Thyroid autoantibodies	2	7	7	31.8	18	33.3	27	27.3	*P* < 0.03
TSH	0.87 ± 0.07		2.99 ± 0.7		3.28 ± 1.9				*P* < 0.05

DKA: diabetic ketoacidosis, FH: family history, T1DM: type 1 diabetes mellitus, T2DM: type 1 diabetes mellitus, TSH: thyroid stimulating hormone.

**Table 2:** Distribution and correlation of the main clinical symptoms preceding diagnosis and the different patients age groups.

Symptoms	Age groups (years)			Total number	*P* value
	<2	2–<6	6–12		
Polyuria and Polydipsia	20	22	51	93	NS
	*87% *	*100.0% *	*94.4% *	*93.9% *	
Weight loss	15	21	52	88	NS
	*65.2% *	*95.5% *	*96.3% *	*88.9% *	
Polyphagia	5	5	12	22	NS
	*21.7% *	*22.7% *	*22.2% *	*22.2% *	
Refusal of feeding	3	1	4	8	NS
	*14.3% *	*4.5% *	*7.4% *	*8.1% *	
Abdominal pain	3	9	40	52	*P* < 0.001**
	*13% *	*40.9% *	*74.1% *	*52.5% *	
Vomiting	11	7	23	41	*P* = 0.393
	*47.8% *	*31.8% *	*42.6% *	*41.4% *	
Dehydration	7	2	11	20	NS
	*30.4% *	*9.1% *	*20.4% *	*20.2% *	
Disturbed conscious level	14	9	23	46	*P* = 0.284
	*60.9% *	*40.9% *	*42.6% *	*46.5% *	
Nocturia and nocturnal enuresis	8	18	48	74	*P* < 0.001**
	*34.7% *	*81.8% *	*88.9% *	*74.7% *	
Infection	4	5	6	15	NS
	*17.4% *	*22.7% *	*11.1% *	*15.2% *	

NS: nonsignificant value, **highly significant.

The article "Epidemiological Pattern of Newly Diagnosed Children with Type 1 Diabetes Mellitus, Taif, Saudi Arabia" was retracted in 2016. Reasons: plagiarized text; content taken from a thesis; overlap with other authors' work; concerns about the citations.

N.B: the classic triad; polyuria, polydipsia, and weight loss; are the dominant presenting symptoms in the 3 age groups followed by vomiting and disturbed conscious level in those <2 years, nocturia and nocturnal enuresis in 2–<6 years age group, and abdominal pain, nocturia, and nocturnal enuresis in the 6–12 years age group.

**Table 3:** Frequency of diabetic ketoacidosis among the different clinical symptoms and signs.

Symptoms/signs	Mode of presentations				*P* value
	Mild DKA	Moderate to severe DKA	Total number of patients with DKA	Total number of children with symptom	
Classic triad	0	8	8	8	*P* < 0.05*
	0.0	100%	100%	100%	
Dehydration	0	17	17	20	*P* < 0.05*
	0.0	100%	85%	100%	
Vomiting	7	32	39	41	*P* < 0.001**
	18%	82.1%	95.1%	100%	
Abdominal pain	13	31	44	52	*P* < 0.01*
	29.5%	70.5%	84.6%	100%	

DKA: diabetic ketoacidosis, *significant, **highly significant.

N.B: most children with DKA whatever the degree of severity presented with abdominal pain and vomiting. Dehydration was present in 100% of those with moderate to severe DKA.

**Table 4:** Implication of different risk factors on the severity of presentation.

Points of comparison	Hyperglycemia		Mild DKA		Moderate-severe DKA		Total		*P* value
	No.	%	No.	%	No.	%	No.	%	
	20	20.2	28	28.3	51	51.5	99	100	
District									
Urban	11	27.5	10	25	19	47.5	40	40	*P* > 0.05
Rural	9	15.3	18	30.5	32	54.2	59	60	
Symptom duration	12 ± 7.6		14 ± 9.5		15 ± 8.6		—		*P* > 0.05
Type of feeding									
Breastfeeding	5	26.3	2	10.5	12	63.2	19	19.2	*P* < 0.05
Cow's milk	16	20.0	27	33.7	37	46.3	80	80.8	
<3 months	6	21.4	7	25.0	15	53.6	28	28.3	
3–6 months	2	8.3	13	54.2	9	37.5	24	24.2	
>6 months	8	28.6	7	25	13	46.4	28	28.3	
Positive family history of DM	17	85	23	82.1	38	74.5	78	78.8	*P* > 0.05

No.: number, DM: diabetes mellitus, DKA: diabetic ketoacidosis.

**Table 5:** Correlation of C-peptide and TSH levels to patients and controls.

Point of comparison	Controls						Patients						*P*-value
	No.	Mean	Std. deviation	Median	Min.	Max.	No.	Mean	Std. deviation	Median	Min.	Max.	
Fasting C-peptide (ng/mL)	110	1.28	0.38	1.30	0.80	1.80	99	1.07	0.66	0.87	0.25	3.80	*P* < 0.001**
TSH *μ*IU/mL	110	3.11	1.60	3.60	0.80	5.30	99	2.38	1.71	2.65	0.80	6.20	0.058

No.: number; Std.: standard; Min.: minimum; Max.: maximum; **highly significant.
